# Texture Analysis in the Assessment of Rectal Cancer: Comparison of T2WI and Diffusion-Weighted Imaging

**DOI:** 10.1155/2021/9976440

**Published:** 2021-09-15

**Authors:** Ming Li, Xiaodan Xu, Pengjiang Qian, Heng Jiang, Jianlong Jiang, Jinbing Sun, Zhihua Lu

**Affiliations:** ^1^Department of General Surgery, Changshu No. 1 People's Hospital, Changshu, 215500 Jiangsu Province, China; ^2^Department of Gastroenterology, Changshu No. 1 People's Hospital, Changshu, 215500 Jiangsu Province, China; ^3^School of Artificial Intelligence and Computer Science, Jiangnan University, Wuxi, 214122 Jiangsu Province, China; ^4^Department of Radiology, Changshu No. 1 People's Hospital, Changshu, 215500 Jiangsu Province, China

## Abstract

Texture analysis (TA) techniques derived from T2-weighted imaging (T2WI) and apparent diffusion coefficient (ADC) maps of rectal cancer can both achieve good diagnosis performance. This study was to compare TA from T2WI and ADC maps between different pathological T and N stages to confirm which TA analysis is better in diagnosis performance. 146 patients were enrolled in this study. Tumor TA was performed on every patient's T2WI and ADC maps, respectively; then, skewness, kurtosis, uniformity, entropy, energy, inertia, and correlation were calculated. Our results demonstrated that those significant different parameters derived from T2WI had better diagnostic performance than those from ADC maps in differentiating pT3b-4 and pN1-2 stage tumors. In particular, the energy derived from T2WI was an optimal parameter for diagnostic efficiency. High-resolution T2WI plays a key point in the local stage of rectal cancer; thus, TA derived from T2WI may be a more useful tool to aid radiologists and surgeons in selecting treatment.

## 1. Introduction

The incidence and mortality of colorectal cancer in China have maintained an upward trend, which ranks third and fifth among all malignant tumors. Among them, rectal cancer accounts for half of colorectal cancer in China. [1].

Pathological T and N stages of rectal cancer were important prognostic factors affecting patients [2]. The patients of rectal cancer with lymph node metastasis require neoadjuvant chemotherapy. pT1-2 stage patients do not require neoadjuvant chemotherapy due to a low recurrence rate; conversely, pT3-4 stage patients need neoadjuvant chemotherapy [3, 4]. The prognosis of pT3 stage rectal cancer varies greatly based on extramural depth (EMD) of tumor invasion [5]. The 5 mm cutoff of EMD has been determined to be the most discriminating and simple to use in clinical practice regardless of differences in overall survival and local recurrence [5–7]. Therefore, an accurate preoperative evaluation is essential because individualized treatment measures are required for different local staging patients.

Diffusion-weighted imaging (DWI) could improve contrast between the lesion and normal tissue, which could improve the accuracy of rectal cancer detection. Compared with T2WI alone, T2WI combined with DWI has the best accuracy and specificity for the diagnosis of rectal cancer; moreover, that can improve accuracy of rectal cancer staging [8, 9].

Texture analysis (TA), as a new image postprocessing technology, can quantitatively describe tissue heterogeneity in medical images. About rectal cancer, there are many TA studies involved on T2WI and ADC maps. The study of Yang et al. [10] reported that T2WI histogram parameters could differentiate the positive and negative lymph node. TA derived from T2WI can be used for prediction of the rectal cancer T stage. [11]. In addition, our previous research results showed that TA from ADC maps could predict the local stage of rectal cancer [12].

In the present study, we investigated to compare TA from T2WI and ADC maps between different pathological T and N stages and to evaluate diagnostic performance to further confirm which TA analysis is better in diagnosis performance.

## 2. Materials and Methods

### 2.1. Patients

This retrospective study was approved by the Institutional Review Board of Changshu Hospital of Soochow University. As this study has retrospective nature, requirements for written informed consent were waived. Inclusion criteria were (1) biopsy-proven nonmucinous adenocarcinoma and (2) the complete pathological T and N stage report. Exclusion criteria were (1) motion artifacts and magnetic sensitive artifacts affecting image quality and (2) treatment with preoperative chemotherapy or radiotherapy.

Finally, 146 patients were enrolled in the final study between October 2016 and October 2020.

### 2.2. MRI

All MRI examinations were performed on 3.0 T scanner (Intera Achieva TX, Philips Medical System) using a phased-array surface coil.

MR sequences included sagittal, oblique axial (perpendicular to the tumor axis), and oblique coronal (parallel to the tumor axis) T2WI and oblique axial DWI (Table 1). The position and scanning parameters of oblique axial DWI were consistent with oblique axial T2WI. The ADC map is automatically generated by DWI with a *b* value of 0 and 1000 s/mm^2^.

### 2.3. Textural Feature Calculation

TA was performed on axial T2WI and ADC maps, respectively, using in-house software (Omni-Kinetics, GE Healthcare) by two authors (Zhihua Lu and Ming Li). The regions of interest (ROIs) involve as much tumor tissue as possible on the largest tumor slice, excluding necrosis, cysts, and gas (Figures 1 and 2). Then, texture features based on T2WI and ADC maps were calculated automatically. The seven texture features that we chose included skewness, kurtosis, and uniformity (first-order statistics) and entropy, energy, inertia, and correlation (second-order statistics).

### 2.4. Histopathologic Analysis

A pathological T (pT) and N (pN) staging report was performed based on the eighth edition of the American Joint Committee on Cancer (AJCC 8th) [13]. The histopathological report of local T and N staging was referred to as the gold standard in this study.

### 2.5. Statistical Analysis

First, the Kolmogorov-Smirnov test was used; data were presented as mean ± standard deviation or median ± interquartile range. To assess the difference of texture parameters between pT1-3a vs. pT3b-4 stage and pN0 vs. pN1-2 stage from the T2WI and ADC maps, the *t*-test or Mann-Whitney *U* test was performed. Subsequent receiver operating characteristic (ROC) curve analysis was performed with those significant different parameters from the T2WI and ADC maps. The correlations between those significant different parameters from the T2WI and ADC maps and pathological T and N stages were used by the Spearman analysis. Intraclass correlation coefficients (ICCs) were calculated for interobserver agreements. SPSS and MedCalc software was used for statistical analysis. The significant level was set as *p* value ≤ 0.05.

## 3. Results

### 3.1. Clinical and Pathological Findings

146 patients comprised 86 males (41-89 years; median, 68 years) and 60 females (41-84 years; median, 67 years). Detailed clinical and pathological data are listed in Table 2. According to the design of this study, 70 patients were grouped as pT1-3a and 76 patients were grouped as pT3b-4. 91 patients were grouped as pN0, and 55 patients were grouped as pN1-2.

### 3.2. Texture Parameters in Differentiating pT1-3a and pT3b-4 Stages

On T2WI, the pT3b-4 stage tumor demonstrated significantly higher kurtosis and entropy and lower energy than the pT1-3a stage tumor (all *p* < 0.05, Table 3). On the ADC map, the pT3b-4 stage tumor demonstrated significantly higher skewness, kurtosis, and entropy than the pT1-3a stage tumor (all *p* < 0.05). No significant differences were found in other TA parameters between different T stages. The results of ICCs are shown in Table 3.

### 3.3. Texture Parameters in Differentiating pN0 and pN1-2 Stages

On T2WI, the pN1-2 stage tumor demonstrated significantly higher skewness and entropy and lower energy than the pN0 stage tumor (all *p* < 0.05, Table 4). On the ADC map, the pN1-2 stage tumor demonstrated significantly higher skewness and kurtosis than the pN0 stage tumor (all *p* < 0.05). No significant differences were found in other TA parameters between different N stages. The results of ICCs are shown in Table 4.

### 3.4. Performance of Texture Parameters to Distinguish the pT3b-4 and pN1-2 Stages

For differentiating pT3b-4 from pT1-3a stage tumors, energy derived from T2WI had the largest AUC (79.3%). Kurtosis derived from the ADC map had the largest AUC (61.8%) (Table 5, Figure 3). Furthermore, energy derived from T2WI showed a better correlation with the pathological T stage (*R*_s_ = −0.494) than kurtosis derived from ADC maps (Table 6).

For differentiating pN1-2 from pN0 stage tumors, energy derived from T2WI had the largest AUC (71.3%). Skewness derived from ADC maps had the largest AUC (61.8%) (Figure 4). Furthermore, energy derived from T2WI showed a better correlation with the pathological N stage (*R*_s_ = −0.359) than skewness derived from ADC maps (Table 6).

## 4. Discussion

The present study showed that kurtosis, energy, and entropy from T2WI and skewness, kurtosis, and entropy from ADC maps could significantly differentiate pT1-3a and pT3b-4 stages. In addition, we found that skewness, energy, and entropy from T2WI and skewness and kurtosis from ADC maps could significantly differentiate pN0 and pN1-2 stages. Among the aforementioned significant different parameters, those parameters derived from T2WI had higher AUC differentiating pT3b-4 and pN1-2 stage tumors than those derived from ADC maps. Furthermore, those parameters derived from T2WI showed a better correlation with pathological T and N stages than those derived from ADC maps. The results indicate that the diagnostic performance of TA parameters derived from T2WI was better than that derived from ADC maps.

High-resolution T2WI plays a key point in the local stage of rectal cancer. In recent years, some studies applied TA derived from T2WI in order to improve the preoperative stage and predict prognostic factors of rectal cancer [10, 11, 14]. In our study, the pT3b-4 stage tumor demonstrated higher kurtosis and entropy and lower energy than the pT1-3a stage tumor. In addition, the pN1-2 stage tumor demonstrated higher skewness and entropy and lower energy than the pN0 stage tumor. Theoretically, higher entropy and lower energy reflect higher heterogeneity of the lesion [15]. This may interpret our results. Yang et al. [10] have reported that the lymph node-positive group had a significant lower energy and higher entropy than the lymph node-negative group.

DWI could improve contrast between the lesion and normal tissue. It has been widely used in preoperative imaging of rectal cancer because T2WI combined with DWI can improve the accuracy of rectal cancer staging [8]. Our previous research and other studies have shown that the ADC value estimated from DWI was related to tumor aggressiveness [16–18]. TA parameters derived from ADC maps were more sensitive and reliable markers for the accurate operative stage and evaluate the efficacy to treatment in rectal cancer [12, 19]. In our study, the pT3b-4 stage tumor demonstrated higher skewness, kurtosis, and entropy than the pT1-3a stage tumor. In addition, the pN1-2 stage tumor demonstrated higher skewness and kurtosis than the pN0 stage tumor. Higher value of skewness and kurtosis reflects more complexity and heterogeneity in tumors. Our result concluded that skewness and kurtosis derived from ADC maps as imaging biomarkers might be differentiating the positive lymph node of rectal cancer.

ROC curves showed that significant different parameters derived from T2WI had higher AUC differentiating pT3b-4 and pN1-2 stage tumors than those derived from ADC maps. Energy was shown to be the best performance in predicting pT3b-4 and pN1-2 stage tumors among TA parameters with yielding AUC of 79.3% and 71.3%, respectively. Furthermore, the Spearman correlation analysis showed that energy derived from T2WI had the better correlation with pathological T and N stages than parameters derived from the ADC map. Therefore, our results indicated that the diagnostic performance of TA parameters derived from T2WI was better than that derived from ADC maps. The reason may be that high-resolution T2WI can reflect much more details in the image of the lesion. In addition, T2WI is the preferred sequence for the preoperative stage of rectal cancer. Thus, TA derived from T2WI may be a more useful tool to aid radiologists and surgeons in selecting treatment.

There are some limitations. First, rectal cancer often grows infiltrating along the bowel wall. Lesions and normal bowel walls are often unclear; then, the measurement cannot accurately delineate the entire tumor. So, the measurement in our study was performed on a single slice of the largest tumor slice. Second, we evaluated seven TA parameters in our study because these parameters have been proven by previous studies to be related to the heterogeneity of the disease. No other more parameters were included for the group study. Third, we only included pathological T and N stage as the grouping standard. More prognostic factors should be included in the later period for further research.

In conclusion, our study showed that the diagnostic performance of TA parameters derived from T2WI was better than that derived from ADC maps. In particular, the energy derived from T2WI was the optimal parameter for diagnostic efficiency. Thus, TA derived from T2WI may be a more useful tool to aid radiologists and surgeons in selecting treatment.

## Figures and Tables

**Figure 1:** Example image for delineating a rectal lesion on T2WI.

**Figure 2:** Example image for delineating a rectal lesion tumor edge on the ADC map.

**Figure 3:** The ROC map of texture parameters in differentiating pT3b-4 from the pT1-3a stage.

**Figure 4:** The ROC map of texture parameters in differentiating pN1-2 from the pN0 stage.

**Table 1:** MRI sequences.

MRI sequence	TR (ms)	TE (ms)	TSE factor	Slice thickness (mm)	Gap (mm)	FOV (cm)	Matrix	NSA	*b*-value
Sagittal T2WI	3577	70	20	3	0	24 × 24 × 7.2	300 × 266	3	—
Coronal T2WI	3000	75	18	2	0	18 × 18 × 0.4	300 × 218	3	—
Axial T2WI	3000	75	18	3	0	18 × 18 × 7.2	368 × 273	3	—
DWI	2750	76	—	3	0	22 × 22 × 7.2	112 × 108	2	0, 1000

TR: repetition time; TE: echo time; TSE: turbo spin echo; FOV: field of view; NSA: number of signal averaged.

**Table 2:** Clinical and pathological data of patients.

Characteristics	No. of patients (*n* = 146)
Gender	
Male	86
Female	60
Tumor location	
Upper rectum	55
Middle rectum	66
Low rectum	25
Differentiated grade	
Well differentiated	28
Moderately differentiated	67
Poorly differentiated	51
Pathological T stage	
T1	8
T2	37
T3a	25
T3b	54
T3c	17
T4	5
Pathological N stage	
N0	91
N1	40
N2	15

**Table 3:** Texture parameters between the pT1-3a and pT3b-4 stages.

Texture parameters	pT1-3a (*n* = 70)	pT3b-4 (*n* = 76)	*p* value	ICC
T2WI				
Skewness	0.785 ± 0.397	0.871 ± 0.384	0.185	0.863
Kurtosis	1.109 ± 0.425	1.378 ± 0.593	0.002	0.885
Energy (×10^−3^)	0.685 (0.580, 0.871)	0.515 (0.452, 0.605)	<0.001	0.847
Entropy	9.226 (8.480, 9.488)	9.590 (9.342, 9.869)	<0.001	0.913
Uniformity	0.812 ± 0.068	0.798 ± 0.073	0.228	0.905
Inertia	159.572 (126.822, 195.283)	163.749 (125.463, 203.394)	0.738	0.865
Correlation (×10^−3^)	1.358 ± 0.470	1.304 ± 0.502	0.508	0.886
ADC				
Skewness	0.382 ± 0.311	0.516 ± 0.360	0.018	0.838
Kurtosis	0.661 ± 0.375	0.809 ± 0.390	0.020	0.875
Energy (×10^−3^)	0.949 (0.625, 0.693)	0.690 (0.583, 1.445)	0.102	0.912
Entropy	9.672 ± 1.203	10.093 ± 1.235	0.039	0.903
Uniformity	0.761 ± 0.057	0.769 ± 0.070	0.502	0.887
Inertia	922.235 (621.034, 1189.230)	737.177 (520.237, 1060.946)	0.086	0.866
Correlation (×10^−3^)	0.448 (0.349, 0.638)	0.482 (0.384, 0.641)	0.267	0.903

**Table 4:** Texture parameters between the pN0 and pN1-2 stages.

Texture parameters	pN0 (*n* = 91)	pN1-2 (*n* = 55)	*p* value	ICC
T2WI				
Skewness	0.763 ± 0.380	0.940 ± 0.389	0.007	0.852
Kurtosis	1.253 ± 0.552	1.243 ± 0.510	0.911	0.856
Energy (×10^−3^)	0.639 (0.530, 0.786)	0.516 (0.437, 0.613)	<0.001	0.867
Entropy	9.342 (8.788, 9.662)	9.537 (9.135, 9.773)	0.039	0.883
Uniformity	0.810 ± 0.064	0.797 ± 0.081	0.333	0.915
Inertia	163.749 (125.463, 203.394)	157.387 (119.347, 184.395)	0.186	0.856
Correlation (×10^−3^)	1.341 ± 0.473	1.312 ± 0.510	0.729	0.863
ADC				
Skewness	0.403 ± 0.283	0.532 ± 0.414	0.045	0.878
Kurtosis	0.682 ± 0.346	0.832 ± 0.437	0.033	0.863
Energy (×10^−3^)	0.832 (0.589, 1.493)	0.710 (0.592, 1.503)	0.747	0.902
Entropy	9.863 ± 1.212	9.938 ± 1.278	0.722	0.893
Uniformity	0.762 ± 0.067	0.771 ± 0.060	0.392	0.907
Inertia	830.845 (529.492, 1116.510)	918.167 (593.935, 1180.040)	0.202	0.916
Correlation (×10^−3^)	0.484 (0.377, 0.734)	0.458 (0.373, 0.637)	0.330	0.905

**Table 5:** Performance of texture parameters to discriminate high-stage tumors.

Parameters	AUC	*p* value	95% CI	Sensitivity (%)	Specificity (%)	Cutoff value
Discriminate pT3b-4 stage						
T2-kurtosis	0.638	0.0028	0.555, 0.716	53.9	75.7	>1.332
T2-energy	0.793	<0.0001	0.718, 0.856	60.5	87.1	≤0.528
T2-entropy	0.743	<0.0001	0.664, 0.811	76.3	64.3	>9.329
A-skewness	0.605	0.0248	0.521, 0.685	30.3	91.4	>0.730
A-kurtosis	0.618	0.0121	0.534, 0.697	50.0	77.1	>0.818
A-entropy	0.602	0.0292	0.518, 0.682	75.0	42.9	>9.395
Discriminate pN1-2 stage						
T2-skewness	0.640	0.0029	0.556, 0.718	70.9	54.9	>0.729
T2-energy	0.713	<0.0001	0.632, 0.784	67.3	73.6	≤0.547
T2-entropy	0.602	0.0313	0.518, 0.682	72.7	48.4	>9.288
A-skewness	0.618	0.0243	0.535, 0.698	40.0	90.1	>0.729
A-kurtosis	0.601	0.0489	0.516, 0.681	29.1	93.4	>1.219

Notes: T2-: texture parameters from the T2WI map; A-: texture parameters from the ADC map; CI: confidence interval; AUC: area under the curve.

**Table 6:** Correlations between significant different parameters from the T2WI and ADC maps and pathological T and N stages.

Parameters	Pathological T stage		Parameters	Pathological N stage	
	*R*_s_	*p* value		*R*_s_	*p* value
T2-kurtosis	0.266	0.001	T2-skewness	0.229	0.005
T2-energy	-0.494	<0.001	T2-energy	-0.359	<0.001
T2-entropy	0.445	<0.001	T2-entropy	0.175	0.035
A-skewness	0.199	0.016	A-skewness	0.196	0.018
A-kurtosis	0.235	0.004	A-kurtosis	0.168	0.043
A-entropy	0.221	0.007			

Notes: T2-: texture parameters from the T2WI map; A-: texture parameters from the ADC map.

## Data Availability

The data used to support the findings of this study are available from the corresponding author upon request.
